# Fine-scale visualizing the hierarchical structure of mouse biliary tree with fluorescence microscopy method

**DOI:** 10.1042/BSR20193757

**Published:** 2020-05-12

**Authors:** Yuwei Chen, Lin Bai, Yongjie Zhou, Xiaoyun Zhang, Jie Zhang, Yujun Shi

**Affiliations:** 1 Laboratory of Pathology, Key Laboratory of Transplant Engineering and Immunology, NHC, West China Hospital, Sichuan University, Chengdu 610041, China; 2 Research Core Facility, West China Hospital, Sichuan University, Chengdu 610041, China; 3 Department of Liver and Vascular Surgery, West China Hospital, Sichuan University, Chengdu 610041, China; 4 Department of Pathology, West China Hospital, Sichuan University, Chengdu 610041, China

**Keywords:** Biliary tract, Confocal microscope, Fluorescence imaging

## Abstract

The liver is a vital organ and the hepatic lobule serves as the most basic structural and functional unit which is mainly assembled with parenchymal cells including hepatocytes and biliary epithelial cells. The continuous tubular arrangement of biliary cells which constitutes the biliary tracts is critical for liver function, however, the biliary tracts are often disrupted in many liver diseases such as cirrhosis and some congenital disorders. Visualization of the biliary tracts in fine-scale and three-dimension will help to understanding the structure basis of these liver diseases. In the present study, we established several biliary tract injury mouse models by diet feeding, surgery or genetic modification. The cytoplasm and nuclei of the parenchymal cells were marked by active uptake of fluorescent dyes Rhodamine B (red) and Hoechst (blue), respectively. After the removal of liver *en bloc*, the biliary tracts were retrogradely perfused with green fluorescent dye, fluorescein isothiocyanate (FITC). The liver was then observed under confocal microscopy. The fine-scale and three-dimensional (3D) structure of the whole biliary tree, particularly the network of the end-terminal bile canaliculi and neighboring hepatocytes were clearly visualized. The biliary tracts displayed clear distinct characteristics in normal liver and diseased liver models. Taken together, we have developed a simple and repeatable imaging method to visualize the fine-scale and hierarchical architecture of the biliary tracts spreading in the mouse liver.

## Introduction

Liver is a highly organized organ and filled with intrahepatic biliary tracts. The hierarchical and well-arranged structure of biliary tracts are pivotal for liver function. The biliary tree is an intricate three-dimensional (3D) network of tubular conduits with various sizes and properties, which is formed mainly by cholangiocytes. The smallest biliary channels are the bile canaliculi which are composed of specializations of the apical membrane of two or more adjacent hepatocytes rather than cholangiocytes [1]. The bile canaliculi converge into Canals of Hering at the edge of hepatic lobule, and drain into septal and interlobular bile ducts which extend into extrahepatic bile ducts [2]. Bile is synthesized by hepatocytes and primarily secreted into bile canaliculi, reabsorbed and modified by cholangiocytes, and then stored in gall bladder, which is drained into duodenum after meals to promote the digestion and absorption of fat [3]. Pathologically, certain conditions often preferentially involve specific portions or segments of the biliary tracts. For example, primary biliary cirrhosis results in destruction that is limited in interlobular and septal bile ducts [4]. In contrast, intrahepatic cholestasis induced by drugs seems to affect the cholangiocytes principally that distribute in terminal bile ducts [5]. Thus, exploration of the entire alteration of the whole biliary tree, especially tiny bile canaliculi among hepatocytes, means great significance.

Many studies have been carried out to visualize the biliary tracts in small animals, however, there are barely few methods that can reach this goal. X-ray and micro-CT scanning are the original ways used to measure the biliary tree, almost with suboptimal spatial resolution of distal biliary ducts. Traditional two-dimensional methods, such as immunohistochemistry (IHC), can only exhibit the cross-section of the 3D structures, and the direction and the complete structure of biliary tree remains elusive [6]. Takashima et al. [7] performed the 3D structural reconstruction based on the images of immunostaining serial-cross sections. However, they required continuous sections of the entire liver to reconstruct the biliary tract and professional computer analysis, which is time-consuming and laborious. Afterward, Sparks et al. initially proposed a method, resin casting together with tissue clearance, to preserve the broad biliary architecture [8–10]. The major disadvantage of resin casting is the damage to the surrounding liver parenchyma. In addition, they were unable to see the fine structures of the bile ducts, such as the Canals of Hering or the bile canaliculi. Based on resin casting, Itoh et al. developed a simpler way to illustrate bile ducts, with only ink retrograded injection into common bile duct [11,12]. However, all the emerging methods for visualizing the biliary tree are unable to present high-resolution images of the tiny bile canaliculi and their spatial relationship with surrounding hepatocytes. Furthermore, none of these strategies are potential to maintain the liver tissue for further examination.

In the present study, we proposed an innovative approach to visualize the panoramic view of the biliary tree by staining the parenchymal cells and filling the biliary tracts with different fluorescent dyes. Then the liver was observed *en bloc* under confocal microscopy. With this novel approach, we succeeded in revealing the fine-scale and hierarchical architecture of biliary tract spreading in the mouse liver and the characteristics of the biliary architecture in three types of injury mouse models.

## Materials and methods

### Animals and liver injury models

All animal experiments were approved by the Institutional Animal Care and Use Committee of the Traditional Chinese Medicine National Center (Chengdu, China) (Protocol: IACUC-2012001C). All animals were maintained under standard specific pathogen-free conditions in the Experimental Animal Center of Sichuan University, China (Animal License No. SYXK(Chuan)2018-119), where the animal work took place. Adult wild-type C57BL/6J mice aged 6–8 weeks were purchased from a commercial supplier (Dashuo Experiment Animal Co. Ltd, Chengdu, China), and PKHD1^−/−^ transgenic mice were a kind gift from Professor Zhou (Sichuan University, China). For biliary injury models, DDC mice were fed 0.1% of 3,5-diethoxycarbonyl-1,4-dihydrocollidine (DDC)-containing diet (Merk–Sigma; Darmstadt, Germany) for 1 month. A surgery of bile duct ligation (BDL) mouse model was constructed by ligating the common bile duct for 10 days. PKHD^−/−^ mice, serving as a model of polycystic liver, were bred under normal conditions for 11–12 months.

### Visualization of the biliary tree

Rhodamine B (Sigma, Cat#230162) is a cell-permeant orange-red fluorescent dye with excitation wavelength of 570 nm and emission wavelength of 590 nm. Hoechst (excitation wavelength: 345 nm; emission wavelength: 478 nm) (Thermo, Cat#H1399) is a perfect material to mark living cell nucleus *in vivo*. Both dyes can be observed in the liver after intraperitoneal injection, and the cytoplasm and nuclei of the liver cells are dyed with orange red and bright blue, respectively. Fluorescein isothiocyanate (FITC, excitation wavelength: 494 nm; emission wavelength: 518 nm) (Sigma, Cat#74817), a common green fluorescent reagent is suitable for the visualization of the biliary tree for biological research, because of its high absorptivity, excellent fluorescence quantum yield and good water solubility. In the present study, the biliary tracts were retrogradely perfused with FITC and the biliary tree exhibited green fluorescence under confocal microscope. Therefore, the hepatocytes, biliary cells and bile ducts were marked with three contrasting fluorescent dyes.

The experimental procedures are present in details in Figure 1: the mixed fluorescent dyes containing Hoechst (1.5 mg/ml) and Rhodamine B (2.5 mg/ml) were intraperitoneally injected at 4 ml/kg body weight. The mixed dyes were transported to the liver through portal system and absorbed by the hepatocytes and cholangiocytes. After 20 min, the mouse was anesthetized by intermittent inhalation of ethyl ether (collected from the Equipment Department of Sichuan University), which was inhaled for 10 s at a time to maintain anesthesia for 5 min. The mouse was fixed in a supine position, the inferior vena cava was cut, the portal vein, hepatic artery and common bile duct were ligated. Then, the whole liver was removed *en bloc* gently without any tear or scratches, and the mouse was killed via cervical dislocation.

**Figure 1:** The detailed experimental procedures to visualize the intrahepatic biliary tract The white arrow shows the mouse liver under confocal imaging.

FITC solution (2 mg/ml) was slowly infused into the intrahepatic biliary tract by retrograde injection from the common bile duct with a needle of 26-gauge and a micro-pump at the speed of 2 ml per hour. The injection was stopped just before the FITC reached the surface and the edge of the liver: excess injection may lead to rupture of hepatic capsule. The optimal amount of fluorescent solution, typically, is approximately 60–100 μl for normal liver in mouse weight at 25–30 g. To avoid circumfluence of FITC solution, the common bile duct was ligated immediately again after removing the needle. The liver was washed with phosphate-buffered saline (PBS) for several times to rinse the scattered dyes on the surface. Last but not least, the whole liver was put on a cover glass for confocal imaging within an hour as shown in Figure 1. Three dimensional confocal images of the liver were obtained on a NIKON A1RMP+ microscope at a resolution of 512 × 512 pixels and image acquisition speed of 30 fps. For the confocal imaging system, the Rhodamine B excitation wavelength was 570 nm, the Hoechst excitation wavelength was 345 nm, and the FITC excitation wavelength was 494 nm, respectively.

### Immunofluorescence and IHC staining

After confocal observation, the liver tissues were collected to estimate the potential for conventional immunofluorescence (IF) and IHC application. Liver tissues are treated in the same way as normal IF and IHC stain. Liver samples were fixed in 10% neutral-buffered formalin for 48 h, and embedded in paraffin. For this purpose, the IF staining of glutamine synthetase (GS, Abcam, Cat #ab49873), β-catenin (Abcam, Cat #ab32572), and CK19 (Abcam, Cat #ab133496) and IHC staining of SOX9 (Abcam, Cat #ab185966) and CK19 were carried out as described previously [13]. The images were captured with fluorescence microscope (Leica DM4000B) and light microscopy (Olympus DP Controller 70), respectively.

## Results

### Successful establishment of different liver injury models

Cholangiocytes are well orchestrated in line to form biliary tract in liver in homeostasis. Upon certain stimulations, such as trauma, drugs or genetic modification(s), the biliary tracts are predisposed to incurring disruption. To corroborate that we can observe the subglobal and fine-scale biliary architecture through our method in pathologic conditions, three mouse models with biliary injury were established. Because the obstruction of common bile duct initiates many pathological events that can lead to biliary dilatation, cholestasis, inflammation and fibrosis, surgery of BDL is one of the most widespread experimental models to induce obstructive cholestatic injury in mice [14–16]. DDC-fed mice have been used widely to study the processes associated with chronic cholangiopathies (e.g., cholestasis and biliary fibrosis) [17–19]. The typical pathological changes of DDC model include extensive injury of biliary epithelial cells, cholestasis, inflammation and active proliferation of bile ducts known as ductular reaction. Meanwhile, PKHD1 deficiency mice (PKHD1^−/−^) which develop spontaneously polycystic kidney and polycystic liver disease were also adopted in the present study [20–22].

Anatomical gross view and histological analysis (Figure 2) proved that injury models were successfully established. The BDL liver was enlarged in size, apparent cholestasis could be seen under the hepatic capsule. H&E staining and CK19 IHC staining showed typical changes of biliary obstruction including the dilated intrahepatic bile duct, multiple focal necrosis, cholestasis and active ductular reaction. The DDC liver displayed dark purple red color and significant enlargement. In histology, DDC liver exhibited a characteristic of chronic cholangitis including biliary epithelial injury, active ductular reaction, bile plug formation and inflammatory infiltration. In PKHD1-deficient liver, many cysts could be seen in gross view. Under microscope, multiple cysts scattered throughout the liver tissue. The cysts were filled with clear fluid and the cyst wall was covered with CK19-positive biliary cells.

**Figure 2:** Gross view and histological examination of the normal liver and three injury models CK19 IHC staining was used to show the biliary epithelium in the livers.

### Visualizing biliary tracts in normal mice

The procedures to visualize the biliary tracts were summarized in Figure 1. After intraperitoneal injection of fluorescent dyes, Rhodamine B and Hoechst, alive hepatocytes and cholangiocytes absorbed the dyes automatically, and the cytoplasm and nuclei were dyed with red and blue color, respectively. The absorbed Rhodamine could subsequently be excreted into the bile and mixed with the retrogradely infused FITC, the bile duct will then be filled with yellow fluorescent liquid under confocal microscope. As shown in Figure 3, the integral intrahepatic biliary tracts, covering most of the liver, were clearly exhibited. The hierarchical structure was also well demonstrated. The intrahepatic biliary system was formed by separate ‘biliary trees’ with their peripheral terminal branches, which were mutually collected or joined with each other.

**Figure 3:** Visualization of the intrahepatic biliary tracts in normal mice (**A**) The hierarchical structures of the intrahepatic biliary tracts were clearly presented. Note that we could see the bile canaliculi and the outline of each hepatocyte in the magnification picture. (**B**) The 3D structure of the biliary tree captured under a confocal microscope. The video showing the 3D biliary tracts was shown in Supplementary Video S1.

The reciprocal relationship between biliary trees, especially the connection between terminal bile ducts and the peripheral hepatocytes was clearly presented. Particularly, we could see the bile canaliculi and the outline of each hepatocyte, which brought a new perspective for understanding the bile duct canaliculi formed by two or more adjacent hepatocytes (Figure 3A). More importantly, taking the advantage of confocal microscope, we were able to capture 50–100 μm in depth liver tissue images for 3D biliary tract reconstruction with 3–5 μm intervals (MV) (Figure 3B and Supplementary Video S1). All these results showed that intrahepatic biliary system was well hierarchically organized and finely distributed in homeostasis.

### The intrahepatic biliary tracts are altered in injury models

BDL and DDC models were adopted to manifest the abnormal biliary tracts in diseased livers. As shown in Figure 4, in BDL liver, the contours of the lumen were extremely irregular. We could make out the definite injury or cholestasis sites caused by obstruction, and see the enlarged bile canaliculi and increasing gap between adjacent hepatocytes. Due to the outflow obstruction of the bile, the liquid in the bile ducts was mixed mainly with excreted Rhodamine and a few retrogradely infused FITC, making the silted bile ducts exhibit pink color. Because of the high pressure in the biliary tracts, the end terminal canaliculi were poorly infused and visualized. Interestingly, we also saw prominent inflammatory cell infiltration of the bile ducts: each enlarged bile duct was circled with a great number of cells, indicated by Hoechst-stained nuclei. It could be judged that these cells are lymphocytes, from the size, distribution and number of the cells. In DDC liver, the hepatocytes were ambiguous. The bile ducts were dilated, discontinuous and the collateral branches were extremely reduced (Figure 4). In PKHD1-deficient mice, multiple cysts indicated by filling defect of all the three fluorescence dyes could be clearly observed (Figure 5).

**Figure 4:** Visualization of the aberrant intrahepatic biliary tracts in BDL and DDC mouse models Note, in BLD liver, white arrowheads show the inflammatory cell infiltration of the bile ducts. White stars indicate the retention of Rhodamine B in the dilated bile ducts, however, we could not clearly distinguish the borderline of the ducts because the gathered lymphocytes are also stained in red with absorbed Rhodamine B. White arrows show the retrogradely perfused FITC in the dilated ducts, and when it mixes with excreted Rhodamine B, a pink color is presented in the merged picture.

**Figure 5:** Visualization of biliary tracts in PKHD-deficient liver The cysts were marked as ‘cs’.

### The liver tissues can be reused after imaging

According to the methods documented previously, livers used for cholangiography are unsuitable for further IF or IHC staining directly. For example, the method of ink injection needs optional clearing of the liver tissue, resin casting even destroys liver parenchyma completely. However, in our method, livers can be immediately imaged after harvested, and all the cells and structures were well preserved, which is distinguished from resin casting or ink injection strategies. In this condition, the livers used after imaging could be reused and the quality met the requirement of IF and IHC staining for both membranous and nuclear proteins detection according to our experiments, as illustrated by GS, CK19, SOX2 and β-catenin staining, respectively (Figure 6).

**Figure 6:** The liver tissue was reused for IF and IHC after imaging (**A**) IF stain for GS, CK19, and β-catenin in the liver tissues after imaging. (**B**) IHC for SOX9 and CK19 in DDC liver tissue after imaging.

## Discussion

There are very little of studies in which the imaging of biliary tract can be seen from macro to micro at the same time as yet. It is clearly necessary to establish a new understanding of the limitations of existing visualization methods. Here, we developed a novel experimental imaging technique that enables to directly visualize the intrahepatic biliary tract in a terrific easy and effective way. We captured the images of the biliary tract and the adaptive changes in normal and pathologic conditions, based on fluorescence, cholangiography and high-resolution confocal microscope imaging. The novel protocol can be implemented to display the 3D structure of the whole biliary trees clearly, particularly the network of the terminal bile canaliculus and neighboring hepatocytes.

Our approach has numerous advantages, which is better than previous reported methods of visualization, including X-ray micro-CT scanning, resin casting and ink retrograde injection [10,12,23]. First of all, our method has a high resolution and we can see the outline of each hepatocyte. The interconnection of the biliary trees, even the relationship between the bile canaliculi and adjacent hepatocytes, at a cell level, are clearly presented. Because canaliculus is a membrane structure composed of specialization of the surface of adjacent hepatocytes, neither the most commonly used resin casting nor the ink method can show this structure [12,24]. At present, besides electron microscopy [25] and IF staining with antibodies such as ZO-1 [26], our method can image the bile canaliculus in a completely new way.

Our experimental method is simple, effective, low cost and time saving. The whole experiment can be completed in an hour without much more procedures compared with other methods. Due to the use of various fluorescent dyes, the whole liver has presented three contrasting fluorescence colors under confocal microscopy. It makes each structure of the liver clearer and the contrast more obvious. More importantly, the 3D reconstruction image can also be acquired. In our experiment, we captured images from 50 to 100 μm in depth with 3–5 μm intervals of liver sections and the 3D view was automatically generated, therefore, we just put the whole liver for confocal imaging to realize the 3D reconstruction. And then, if necessary, with a life support system, we can visualize the biliary tree architecture in a living mouse, even the entire dynamic process of dye absorption and excretion, which is much better than magnetic resonance cholangiography (MRC) and near-infrared (NIR) [27,28]. Furthermore, this method can also be applied *in vivo*. We have developed an *in vivo* lineage tracing strategy based on Cre-loxp system to observe the target cells in living mouse [29]. Similarly, by taking advantage of a transgenic strains with fluorescent reporters and two-photon microscopy, Huang et al. recently reported they observed the development of mouse embryos intravitally [30].

The integrity of the liver and the structure of the bile ducts remain unchanged after visualizing the biliary tract. Therefore, another advantage of this approach is that the liver tissues can be reused for further examination, such as IF or IHC staining. Because the cells are all alive and the fluorescent dyes can be excreted from the cells spontaneously, the use of fluorescent dyes will not interfere with further processes. We can even extract protein and nuclear acid qualified for immunoblotting and sequencing if the entire procedure could be finished within 1 h. The method is sample saving, which would be more valuable particularly when the sample is precious.

One of the most notable limitations in our method is that it is difficult to control the total amount of perfused solution accurately, which may result in insufficient or excessive perfusion. Using a microinfusion pump, we can perfuse the whole liver evenly and stop the pump when the dye reaches capsule, however, this is not very accurate and objective. Most of all, a confocal microscopy is essential, which is still an expensive equipment.

In summary, the present study demonstrates a novel imaging method to visualize the fine-scale and hierarchical architecture of the biliary tracts. The protocol generates a deeper understanding of the terminal canaliculus. Furthermore, with the development of microscope imaging technology, more high-resolution pictures can be acquired, which could greatly facilitate biliary tract imaging in basic animal study.

## Supplementary Material

Supplementary Video S1

## Abbreviations

BDL: bile duct ligation
DDC: 3,5-diethoxycarbonyl-1,4-dihydrocollidine
FITC: fluorescein isothiocyanate
GS: glutamine synthetase
H&E: hematoxylin-eosin staining
IF: immunofluorescence
IHC: immunohistochemistry
ZO-1: zonula occludens-1
3D: three-dimensional
